# Mitophagy: A Potential Target for Pressure Overload-Induced Cardiac Remodelling

**DOI:** 10.1155/2022/2849985

**Published:** 2022-09-27

**Authors:** Ruochen Shao, Junli Li, Tianyi Qu, Yanbiao Liao, Mao Chen

**Affiliations:** ^1^Laboratory of Heart Valve Disease, West China Hospital, Sichuan University, 37 Guoxue Street, Chengdu 610064, China; ^2^Department of Cardiology, West China Hospital, Sichuan University, 37 Guoxue Street, Chengdu 610064, China; ^3^Department of Clinical Research Management, West China Hospital, Sichuan University, 37 Guoxue Street, Chengdu 610064, China

## Abstract

The pathological mechanisms underlying cardiac remodelling and cardiac dysfunction caused by pressure overload are poorly understood. Mitochondrial damage and functional dysfunction, including mitochondrial bioenergetic disorder, oxidative stress, and mtDNA damage, contribute to heart injury caused by pressure overload. Mitophagy, an important regulator of mitochondrial homeostasis and function, is triggered by mitochondrial damage and participates in the pathological process of cardiovascular diseases. Recent studies indicate that mitophagy plays a critical role in the pressure overload model, but evidence on the causal relationship between mitophagy abnormality and pressure overload-induced heart injury is inconclusive. This review summarises the mechanism, role, and regulation of mitophagy in the pressure overload model. It also pays special attention to active compounds that may regulate mitophagy in pressure overload, which provide clues for possible clinical applications.

## 1. Introduction

Pressure overload-induced cardiac dysfunction is a common pathological basis in numerous heart disease, including aortic stenosis and chronic hypertension. Pressure overload induced by TAC has become a classical animal model in rodents to simulate cardiac damage caused by pressure overload in humans [1]. Continuous exposure to increased pressure gradually transforms the initially compensatory response into pathological cardiac remodelling, manifested as increased cardiomyocyte mass, sarcomere rearrangement, extracellular matrix deposition, and immune cell activation, which eventually lead to terminal-stage heart failure [2, 3]. The heart mainly relies on mitochondria to manufacture the energy used for its contractile function; these account for over 30% of the volume of myocardial cells and provide 90% of cellular ATP energy via oxidative phosphorylation and fatty acid oxidation [4]. Mitochondria are also involved in various key cellular processes, such as the regulation of cell proliferation and apoptosis, maintenance of calcium homeostasis, and communication and functional coordination with lysosomes, the endoplasmic reticulum, the nucleus, and other organelles [5, 6]. Therefore, the abnormality of the structure and function of mitochondria in the pressure overload model has been frequently investigated. In vivo and in vitro experiments have confirmed that mitochondria swell and cristae become fragmented and disordered in cardiomyocytes under pressure overload [7, 8]. Mitophagy is a selective autophagy pathway that mediates mitochondrial quality control by scavenging damaged mitochondria and coordinating the dynamic balance between mitochondrial and cellular energy requirements [9] (Figure 1). Although mitophagy has been widely studied in the pressure overload model, the role, regulation, and potential clinical interventions of mitophagy have not been systematically summarised. This review addresses this gap and generalises the problems that remain to be explored.

## 2. Mitochondrial-Related Damage in Pressure Overload Model

### 2.1. Mitochondrial Bioenergetic Disorder

Heart failure caused by pressure overload is accompanied by a decline in mitochondrial respiratory capacity [10]. Morphologically, mitochondrial cristae disorders, decreased cristae density, and mitochondrial swelling occur after pressure overload [11, 12]. Bugger et al. [11] identified that oxidative phosphorylation and fatty acid oxidation proteins are generally downregulated. Griffiths et al. [13] found that the activities of ETC complexes I and II are significantly impaired after TAC, which may be a reasonable explanation for the reduction of ATP production in the hypertrophic myocardium. One mitochondrial proteomic study revealed that metabolism-related ETC proteins account for over half of the mitochondrial proteins that change significantly after TAC and that the subunits of complex I, III, IV, and V are abnormal [14]. Some interventions on the cardiac phenotype of pressure overload can be attributed to improving mitochondrial respiratory function. MitoQ is a mitochondrial antioxidant that restores the potential of interfibrillar mitochondria for ATP production and mitochondrial respiratory function. MitoQ treatment has been shown to reduce cardiac hypertrophy caused by pressure overload through this mechanism [15]. AMS alleviates myocardial hypertrophy and fibrosis after TAC. At the same time, AMS has been reported to increase the expression and activity of complex I, II, III, IV, V, and oxidative phosphorylation-related proteins and to increase mitochondrial membrane potential and mitochondrial oxygen consumption rate [16].

### 2.2. Oxidative Stress

Previous studies have fully proved the role of oxidative stress in cardiac hypertrophy and cardiac dysfunction induced by pressure overload. Oxidative stress occurs when the rate of metabolism or inactivation of ROS and RNS do not match their production rate [17]. Mitochondrial-derived ROS were reported to mediate heart failure induced by volume overload [18]. Subsequently, many experiments have confirmed its negative role in the pressure overload model. ROS can activate various hypertrophy signal pathways, mediate extracellular matrix remodelling by activating matrix metalloproteinase, mediate cardiomyocyte apoptosis, and modify excitation-contraction coupling to induce cardiac hypertrophy due to pressure overload [19, 20]. Intracellular ROS mainly comes from the mitochondrial respiratory chain [21, 22]. Outside mitochondria, NOXs produce O_2_^•-^ by transferring electrons from NADPH to molecular oxygen [23]. In the TAC model, the absence of NOX4 attenuate the production of O_2_^•-^ and alleviates cardiac hypertrophy and cardiac remodelling caused by pressure overload [24]. Shimizu et al. [25] found in the rat heart pressure overload model, mitochondrial BH4 decreased, which mediated the decoupling of NOS3 into monomer to generate O_2_^•-^, and no longer produced the protective NO in the form of a dimer. Superoxide dismutase performs a protective mechanism against oxygen free radicals and converts O_2_^•-^ into H_2_O_2_, which also causes damage to bioactive molecules [26]. O_2_^•-^ can also undergo the Haber-Weiss reaction with existing H_2_O_2_ to produce hydroxyl radicals with more vital oxidation [27]. O_2_^•-^ can also reduce NO to ONOO^−^, thus inhibiting mitochondrial respiratory complex through tyrosine nitration and resulting in both reduced ATP synthesis and cell dysfunction [28]. In human cardiomyocytes, ONOO^−^ induces the nitration of alpha-actinin, resulting in systolic dysfunction [29]. Exposure to ONOO^−^ releases Zn^2+^ from the zinc-thiolate cluster of NOS and destroys the NOS dimer [30]. Targeting oxidative stress has become a hot spot in cardiac remodelling and cardiac dysfunction intervention under pressure overload. Exogenous BH4 supplementation recouples NOS, inhibits ROS, and saves cardiac remodelling after TAC [31, 32]. Murphy et al. [33] suggested that Ffar4 reduces oxidative stress and potentially protects the heart after TAC. Zang et al. [34] revealed that the overexpression of JMJD1A promotes the production of catalase, reduces mitochondrial ROS and total cellular ROS, and inhibits cardiomyocyte hypertrophy.

### 2.3. mtDNA Homeostasis

Human mtDNA is a small amount of closed-loop double-stranded DNA in the mitochondrial matrix. It is responsible for coding 37 genes, including 2 ribosomal subunits, 13 subunits of ETC, and transfer RNA [35]. mtDNA plays an unparalleled role in maintaining mitochondrial function and is associated with various pathological changes of the human myocardium. Ischaemia–reperfusion leads to oxidative damage of mtDNA and reduces its content and transcription levels. Lycopene protects cardiomyocytes from ischaemia–reperfusion injury through its antioxidant properties and the function of preventing the reduction of mitochondrial transcription factor A, which maintains mtDNA stability [36]. mtDNA damage includes (but is not limited to) point mutation and the removal of mtDNA copy number, due to its proximity to ROS production sites, lack of histone protection, and repair dysfunction in specific cases [37]. mtDNA replication is performed by Pol *γ*. Under oxidative stress, Pol *γ* reduces its exonuclease activity, increases mutation, and decreases mtDNA copy number [38]. ROS also induces strand breaks and abasic sites, leading to mtDNA double-strand breaks and degradation [39]. In rat cardiomyocytes, mtDNA damage leads to mitochondrial dysfunction, which further worsens the imbalance of electron transfer and produces ROS, forming a series of vicious cycles [36]. Consistent with these theories, multitudinous studies have detected mtDNA depletion and oxidative damage under pressure overload. Zou et al. [40] found that knockdown of NDUFS1 increases ROS production, downregulates mtDNA content, and develops cardiac hypertrophy under pressure overload. Kuroda et al. [24] observed an increase in mitochondrial DNA content after knockout of NOX4 in mice, with significantly alleviated cardiac hypertrophy and interstitial fibrosis exhibited in response to pressure overload. Twinkle is an integral part of the minimal replication complex of mtDNA and acts as a part of annealing and helicase. It plays a role in mtDNA replication initiation and damage repair [41]. In the pressure overload model, the overexpression of Twinkle increases the copy number of mtDNA and alleviates the deterioration of cardiac function caused by cardiac fibrosis after TAC [42]. In vitro experiments have confirmed that Twinkle can inhibit the TGF-*β*1 signalling pathway [42]. Silymarin is a widely used natural bioactive substance that can increase the concentration of mitochondrial DNA; it prevented cardiac hypertrophy in a rat model of partial abdominal aortic coarctation [43].

## 3. Potential Role of Mitophagy in Pathological Cardiac Remodelling under Pressure Overload

When cells are under the pressure of ROS, mitophagy is activated in a variety of ways. On the one hand, ROS activates mitophagy at the transcriptional level. ROS can activate TIGAR, BINP3/NIX, LC3, P62, and Atg4 to induce autophagy through P53, HIF-1, FOXO3, and Nrf2 pathways [44]. On the other hand, ROS interact with ubiquitin-dependent mitophagy [45]. However, the effect of RNS on Pink1/Parkin remains controversial. NO·free radical-induced S-nitrosylation at Cys568 of Pink1 inhibits its ability to phosphorylate Parkin and reduces Parkin recruitment to mitochondria [46]. S-Nitrosylation of Parkin in Cys323 enhances its E3 ligase activity [47]. The initiation of mitophagy can inhibit the production of ROS in mitochondria to avoid oxidative damage and then inhibit pressure overload-induced myocardial hypertrophy and fibrosis and improve cardiac systolic dysfunction [48]. Mitophagy is also capable of mediating the elimination of damaged mtDNA. In adult drosophila cells, the activation of Pink1/Parkin promotes mitophagy and clears mtDNA, with multiple genes removed or destroyed [49]. ATAD3B was recently identified as a novel mitophagy receptor. ATAD3B is a mitochondrial outer membrane protein that binds to LC3 through its LIR-3 (LC3 interaction region) motif and connects to mtDNA through the ATAD3B–ATAD3BA–mtDNA axis. Under oxidative stress, the heterooligomer of ATAD3B-ATAD3BA decreases, resulting in the exposure of its LIR motif in the cytoplasm, activating mitophagy and eliminating mtDNA mutations that induce oxidative stress [50]. Numerous studies have shown that mitophagy plays an important role in mitochondrial ecology, but mitophagy does not always play a protective role in disease models under unrestricted conditions. Zhang et al. [51] showed that melatonin alleviates cardiac ischaemia–reperfusion injury by activating OPA1-related mitophagy. The deletion of DUSP1 promotes BNIP3-mediated mitophagy and aggravates cardiac dysfunction caused by ischaemia–reperfusion injury [52]. The double-edged sword effect of mitophagy in numerous organs and systems reveals that the regulation and effect of mitophagy are generally related and coordinated. Although there are certain clues, the specific phenotypes caused by mitophagy in different scenarios still need to be examined holistically and dialectically. Fully mobilising active mitophagy while avoiding uncontrolled or maladaptive mitophagy is the key to alleviating cardiac remodelling and cardiac dysfunction caused by pressure overload (Figure 2).

## 4. Regulation of Mitophagy during Cardiac Pressure Overload

### 4.1. Mitochondrial Dynamics

#### 4.1.1. Mitochondrial Division and Fusion

Mitochondrial division and fusion promote the circulation of matrix components between mitochondria, which is of great significance for maintaining their function [53]. Mitochondrial fusion can dynamically repair reversible damage to parts of mitochondria to form functional elongated organelles. Mitochondrial fission occurs when the mitochondria are irreversibly damaged [54]. MFN1, MFN2, and OPA1 mainly mediate mitochondrial fusion [55]. The C-terminal and redox sensitive cysteine residue residence of MFN1 and MFN2 are located in the IMS of mitochondria, and redox-mediated disulfide modifications within the IMS domain regulate the oligomerization of MFNs [56]. MFNs can form MFN1 isooligomers, MFN2 isooligomers, and MFN1-MFN2 heterooligomers. These three types of complexes cooperate to bind the outer mitochondrial membrane of adjacent mitochondria and mediate outer membrane fusion [57, 58]. Mitochondrial intimal fusion depends on OPA1, which is a member of the GTPase family. It is located on the mitochondrial ridge and is of great significance in maintaining mitochondrial morphology. After OPA1-specific knockout, mitochondrial inner membrane fusion is blocked; mitochondrial cristae disappear and multiple matrix components appear inside, but mitochondrial outer membrane fusion is not affected [59]. Membrane-anchored long-form OPA1 (L-OPA1) is hydrolysed at site S1 or S2 by a group of proteases located in the mitochondrial membrane space, resulting in the loss of OPA1 transmembrane domain and the production of soluble short form OPA1 (S-OPA1) [60]. Using the helical three-dimensional reconstruction technology of freeze electron microscope, Zhang et al. [61] found that s-OPA1 can be divided into three parts: GTPase domain for GTP hydrolysis, STALK region mediating the formation of high polymer assembly state, and EMB domain related to membrane binding. S-OPA1, after GTP*γ*S-binding, makes its arrangement on liposome tubes looser by adjusting its own conformation and assembly mode, which is closely related to the function of OPA1 in inducing mitochondrial intimal fusion [61]. S-OPA1 cooperates with L-OPA1 to catalyse fast and efficient fusion. Equimolar L-OPA1 and S-OPA1 mediate the best pore opening efficiency and pore opening kinetics [62].

Mitochondrial fission is mainly regulated by DRP1 [63]. DRP1 has an N-terminal GTPase domain thought to provide mechanical force, a dynamin-like middle domain, and a GTPase effector domain located in the C-terminal region [64]. DRP1 is recruited to the outer mitochondrial membrane by a variety of resident protein receptors, including FIS1, MFF, MID49, and MID51 [23], and cleaves mitochondria when GTPase decomposes GTP for energy [65]. MFF plays a recruiting role for DRP1 through its 50 residues containing short amino acid repeats [65]. The actual function of some protein receptors remains controversial. According to Oliver et al. [66], FIS1, MID49, and MID51 can recruit DRP1 and promote mitochondrial fission. However, some studies have indicated that overexpression of MID49 and MID51 recruits DRP1 to mitochondria and causes mitochondrial fusion [67, 68]. Knocking down FIS1 in HCT116 cells does not reduce the level of DRP1 localised to mitochondria [69]. In a nutshell, the regulation of DRP1 recruitment and subsequent fission induction is subject to complex regulation.

#### 4.1.2. Interaction between Mitochondrial Dynamics and Mitophagy

There is increasing evidence that mitochondrial dynamics coordinate mitophagy as a coherent mechanism. Gilad et al. [70] found the asymmetric division of mildly damaged mitochondria resulted in a healthy hyperpolarised mitochondrion, while another depolarised mitochondrion was cleared by mitophagy. In MEFs, mitochondrial fusion disorder caused by the knockout of MFN1 and MFN2 inhibits mitophagy during mitochondrial damage and leads to the accumulation of dysfunctional mitochondria [71]. MFN2 can mediate mitophagy as a mitochondrial receptor of Parkin. Pink1-mediated phosphorylation of MFN2 at Thr111 and Ser442 results in Parkin binding activity of MFN2. Functional ablation of these phosphorylation sites by their mutational substitution with Ala abrogates MFN2-Parkin binding, whereas mimicking MFN2 phosphorylation by mutational substitution with Glu confers constitutive Parkin binding [72]. MFN2 knockdown can also lead to impaired autophagy degradation and reduce autophagy flux to inhibit mitophagy. In the heart, MFN2 mediates autophagosome-lysosome fusion by attracting and binding RAB7 to the autophagosome membrane. MFN2-deficient mice were reported to have a large accumulation of autophagosomes in the heart [73]. MFN2 can also connect the endoplasmic reticulum and mitochondria by forming homo- and heterocomplexes with MFN1 or MFN2 on mitochondria through MFN2 at the endoplasmic reticulum [74]. This may indicate that the ER–mitochondrial contact site plays a role in mitophagy and may act as a bridge between mitochondrial dynamics and mitophagy. In the dominantly inherited optic atrophy model, OPA1 has shown negative regulation of mitophagy [75]. However, there is evidence that OPA1 plays a role in promoting mitophagy in the heart. Zhang et al. [51] found that melatonin-mediated mitophagy was inhibited after the knockout of OPA1. According to Xin et al. [76], OPA1 overexpression protects cardiomyocytes against hypoxia-induced damage and enhanced cell viability by inducing mitophagy. DRP1 and its receptors are also involved in mitophagy. BNIP3 is an effective inducer of mitophagy. It induces mitochondrial translocation of DRP1, and the inhibition of DRP1 reduces BNIP3-mediated mitophagy [77]. In the myocardium, DRP1 downregulation induces mitochondrial elongation and the accumulation of damaged mitochondria and inhibits mitophagy [78]. Six amino acid domains between Dnm1 (Drp1, Dnm1 in yeast) 24△ and Dnm1 30△ at the C-terminal of Dnm1 GTPase domain in yeast can bind to ATG11 and mediate mitochondrial degradation through the interaction between ATG32 and ATG11 [79]. By contrast, Song et al. [71] proposed that inhibition of DRP1, thereby inhibiting mitochondrial division, enhances mitochondrial autophagy. Yamashita and Kanki [80] proposed a new Dnm1-independent model of simultaneous mitophagy and mitochondrial division, where the budded portion of the mitochondria is divided simultaneously with phagophore closure. Burman et al. [81] had a similar view that DRP1-mediated mitochondrial division does not affect mitophagy. Instead, it protects healthy mitochondrial domains against elimination by the unchecked Pink1-Parkin activity [81]. After 2 hours of CCCP treatment, the loss of MFF significantly reduced the translocation of Parkin from the cytoplasm to damaged mitochondria and prevented mitochondrial clearance; Parkin ubiquitinated MFF at lysine 251, and the K251r mutant of MFF lost its P62 binding activity [82]. Knockdown of MID49 initiates Parkin translocation after CCCP short-term stimulation, further accelerates the degradation of MFN2 and FIS1 through the UPS pathway, and positively regulates mitophagy [83]. Overexpression of exogenous FIS1 enhances autophagosome production of mitophagy in MEF cells [84]. TBC1D15, a mitochondrial Rab GTPase-activating protein, and its amino acid residues 200–300 directly interact with FIS1 and further promote proper autophagic encapsulation of mitochondria [85]. STX17 is localised to the endoplasmic reticulum and mitochondria and regulates mitochondrial division by determining the localisation and fissionable activity of DRP1 [86]. However, the TPR2 structure of FIS1 can bind to STX17 and negatively regulate STX17-induced mitophagy [87]. In conclusion, various mitochondrial dynamic proteins play important roles in balancing mitophagy. These contradictory data support the complex regulation of mitochondria shaping proteins in mitophagy. The regulation of mitophagy by mitochondrial dynamics is not a simple dichotomous relationship, and different regulatory modes dominate in different cells and models, mediating a variety of effects.

#### 4.1.3. Mitochondrial Dynamics in Pressure Overload Models

Abnormal mitochondrial fission and fusion are the main causes of multiple human diseases [88, 89]. Numerous studies have revealed that mitochondrial dynamics and dynamic-related proteins including MFN2, OPA1, and DRP1 play critical role in pressure overload myocardial hypertrophy. MFN2 was found to be downregulated in both spontaneous hypertension and TAC-induced pressure overload models [90]. In vitro, a decrease of MFN2 was also observed in Ang II-induced cardiomyocyte injury [91]. The binding domain of Mir-17-5p significantly increases after TAC. It complements the 3′-UTR of MFN2 and negatively regulates MFN2 expression. Restoring the MFN2 level can reduce cardiomyocyte hypertrophy caused by Mir-17-5p [92]. Another study on the TAC model found that Mir-106a is able to promote cardiac hypertrophy. In the associated in vitro experiments, MFN2 was proved to be a downstream target inhibited by Mir-106a to play a role in promoting hypertrophy [93]. A recent study confirmed that TAC resulted in more significant ventricular dilation and ventricular dysfunction in OPA1^+/-^ mice [94]. Guo et al. [95] found that fatty acids inhibited L-OPA1 to S-OPA1 transformation by upregulation of YME1L and improved mitochondrial and cardiac function in TAC mice. In mice cardiomyocytes, TNFR2 activation-mediated acetylation of K370 and K383 residues at STAT3 increased STAT3/RelA interaction to activate OPA1 expression and played a protective role in TAC-induced mouse cardiac remodelling [96].

Not only fusion proteins of mitochondria but also fission proteins are reported to participate TAC-induced cardiac dysfunction. Myocardial sections obtained from human heart failure patients showed significantly lower DRP1 phosphorylation at S616 than in normal controls [97]. In mice, the phosphorylation of DRP1 at S616 increased significantly soon after TAC, reflecting the enhancement of mitochondrial fission mediated by DRP1. At the same time, the lysosomal localisation of Mito-Keima increased, reflecting the enhancement of mitophagy. However, TAC suppresses mitophagy after 7 days with the downregulation of phosphorylation of DRP1 at S616, followed by mitochondrial dysfunction [97]. Cardiac-specific heterozygotic knockout of DRP1 was reported to exacerbate pressure overload-induced mitochondrial dysfunction, cardiac hypertrophy, and cardiac dysfunction [97]. However, Ma et al. [98] concluded that excessive mitochondrial division and mitophagy are the causes of mitochondrial structure and function damage after TAC, aerobic exercise, and choline intervention balances mitochondrial fusion and fission, reduces mitophagy, and improves cardiac hypertrophy after TAC. Givvimani et al. [99] improved cardiac dysfunction and ventricular remodelling after TAC, I/R, or LPS treatment using the DRP1 inhibitor Mdivi-1, Dynasore or P110. However, the evidence provided by small molecule inhibitors and gene knockout was not completely consistent. These studies show that although existing research cannot provide irrefutable conclusions, it is undeniable that mitochondrial dynamics are a potentially promising intervention target to provide protection when the heart is exposed to pressure overload injury (Figure 3).

### 4.2. Ubiquitin Pathways (Pink1/Parkin)

According to the available data, Pink1/Parkin-mediated mitophagy has been relatively fully characterised. Pink1 is a Ser/Thr kinase that takes possession of an N-terminal mitochondrial targeting sequence (MTS), *α*-helical transmembrane domain, and conserved Ser/Thr domain, along with the C-terminal regulatory domain [100]. The MTS of Pink1 is recognised by Tom20 and Tom22 and passes through the Tom40 channel [101]. Then, it enters the interior of mitochondria through TIM23 driven by mitochondrial inner membrane potential [101]. Under physiological conditions, mitochondrial processing peptidase cuts the MTS sequence of Pink1 [102], and presenilin-associated rhomboid-like protein cuts the amino acid between Ala-103 and Phe-104 of the transmembrane domain of Pink1 [103], which promotes the translocation of Pink1 precursors into the cytoplasm. Parkin is an E3 ubiquitin ligase composed of a ubiquitin-like domain, a 60-amino acid linker, and zinc finger domains (RING) [104]. Parkin is originally in a state of automatic inhibition. The RING0 domain blocks the Cys431 site in the RING2 domain, and the *α* helix bound to RING1 (reporter element of Parkin) blocks the E2 binding site in the RING1 region [104]. When Parkin is activated by injury, the Parkin conformation changes and exposes its C431 site [105]. Parkin collaborates with E1 activating enzyme together with E2 binding enzyme to promote substrate protein ubiquitination [106]. Pink1 accumulates on the outer mitochondrial membrane when the mitochondrial membrane potential is lost [107], which leads to autophosphorylation at the Ser228 and Ser402 sites of Pink1 and summons Parkin to mitochondria [108]. Parkin ubiquitination is not limited to substrate MOM proteins such as VDAC1, MFN1, and MFN2 [109]. Pink1 phosphorylates the Ser65 residue of Parkin and amplifies its E3 ligase activity under excitation by potential depolarisation of the mitochondrial membrane [110]. Subsequently, they are recognised by a variety of autophagy receptors, such as NDP52, OPTN, and P62, and then expand autophagosomes through the LC3 interaction region [111]. On the other hand, Pink1-mediated mitophagy may not depend on Parkin. In cells lacking Parkin, Pink1 can phosphorylate ubiquitin protein and mobilise OPTN and NDP52 to mitochondria, and then ULK1, DFCP1, and WIPI1 are recruited to initiate autophagy [112]. The preponderance of evidence suggests that pathways targeting Pink1/Parkin exert influences on pressure overload, although the current results show divergences to some extent. There is evidence that the upregulation of Pink/Parkin under pressure overload plays a protective role [113]. Cao et al.'s research provides another perspective: Miro2 mediates mitochondrial communication through mitochondrial nanotube formation, which maintains mitochondrial function and heart function under stress overload [114]. After TAC, increased Parkin degrades Miro2 through the ubiquitination pathway [114]. To sum up, the role of the Pink–Parkin pathway in mediating mitophagy in heart failure induced by pressure overload needs the support of additional research.

### 4.3. Mitophagy Receptor Pathways

#### 4.3.1. BNIP3/NIX

BNIP3 and NIX are proteins with homology to BCL2 in the BH3 domain [115]. BNIP3 and NIX have multiple effects of inducing cell death and mitophagy [115]. BNIP3 acts as an effective inducer of autophagy in a variety of cells, including cardiomyocytes [116]. Six residues in BNIP3 are important for dimerisation. They jointly mediate the formation of BNIP3 dimer by forming inter monomer hydrogen bonds, tandem GXXG motif, and Van der Waals contacts [117]. LC3 binds to the LIR motif in the BNIP3 homodimer to induce mitophagy and endoplasmic reticulum autophagy [118]. Phosphorylation of serine residues 17 and 24 on both sides of BNIP3 LIR promotes its binding to LC3B and GATE-16 [119]. The role of NIX in mitophagy was first found in the process of erythrocyte differentiation and maturation [120]. Subsequently, Sandoval et al. [121] found that NIX induces mitophagy by mediating the reduction of mitochondrial membrane potential. Yang et al. [122] demonstrated that NIX deficiency does not interfere with Parkin's recruitment of mitochondria and recognised that NIX mediates mitophagy independently of Parkin and plays a compensatory role at a low level of Parkin. At present, NIX is defined as a selective mitophagy receiver because its terminal amino acids 3–38 form an LIR sequence and bind to LC3a [123]. NIX-mediated mitophagy requires phosphorylation of NIX Ser81, and NIX S81a mutation cannot bind to LC3a or LC3b [122]. NIX usually appears as a homologous dimer [124] through the important role of glycine 204 and glycine 208 in the transmembrane domain. The dimerised NIX significantly increases the binding percentage of LC3a compared with the NIX monomer [124]. Other studies have confirmed the interaction between Nix and the Pink–Parkin pathway. The C-terminal transmembrane domain of BNIP3 binds to Pink1 and inhibits the cleavage of Pink1, promoting the recruitment of Parkin to mitochondria and mitophagy [125]. The current evidence tends to suggest that BNIP3-mediated mitophagy aggravates the negative effects of pressure. BNIP3/NIX is significantly increased after receiving TAC [126]. Knockout of the RAGE prevented the upregulation of BNIP3 in TAC mice and improved TAC-induced cardiac dysfunction [127]. Another study showed that raloxifene is a novel IL-6 inhibitor that can inhibit IL-6-induced BNIP3 elevation as well as cardiac dysfunction and remodelling caused by pressure overload [128]. In vitro, the stress-related hormone norepinephrine induces the upregulation of NIX in 3T3 cells and promotes the expression of collagen and fibronectin [129]. After being transfected with BNIP3, H9C2 cells show both hypertrophic growth (accompanied by the activation of many upstream pathways related to myocardial hypertrophy) and increases in ANP and BNP [130].

#### 4.3.2. FUNDC1

In terms of receiver mediated mitophagy pathway, MOM-anchored protein FUNDC1 participates in mitophagy but does not affect autophagy. FUNDC1 is anchored to the mitochondrial outer membrane through its C-terminal domain. The N-terminal cytoplasmic region of FUNDC1 contains a Y (18) xxL (21) motif, which is a typical LIR [131]. Phosphorylation of FUNDC1 at Ser17 binds to LC3b Lys49 to activate mitophagy through additional hydrogen bonds; on the other hand, phosphorylated Tyr18 and Ser13 in FUNDC1 significantly hinder their interaction with the hydrophobic pocket and Atg10 of LC3B [132]. Knockdown of FUNDC1 in SH-SY5Y cells does not affect Pink1 translocation or Parkin recruitment, indicating that FUNDC1 was not involved in Pink1/Parkin-dependent mitophagy [133]. FUNDC1 is also associated with mitochondrial dynamics. FUNDC1 is located in MAMs where it binds to IP3R2, which is localised to the endoplasmic reticulum. FUNDC1 maintains the concentration of Ca^2+^ in the cytoplasm through this effect, thus maintaining the expression of FIS1, mitochondrial fission, and mitophagy [134]. FUNDC1 interacts with OPA1 through its lysine 70 (K70), and the K70a mutation, lacking interaction with OPA1, reduces the recruitment of LC3 [135]. Current studies support a protective role of FUNDC1 in the heart. Alpha-lipoic acid (*α*-LA) is a coenzyme present in mitochondria that reduces cardiac hypertrophy induced by pressure overload [136]. Li et al. [137] found that *α*-La increases the expression of Nrf1 by activating ALDH2; Nrf1 directly binds to the 5′ promoter of FUNDC1 to regulate its expression, thus reducing cardiac hypertrophy and myocardial remodelling caused by pressure overload. Therefore, the regulation of FUNDC1 in mitophagy to alleviate the damage caused by stress overload is expected to be extensively explored and utilised.

### 4.4. MCU and Mitochondrial Calcium Homeostasis

Mitochondrial Ca^2+^ homeostasis imbalance is an important feature of heart failure caused by pressure overload; mitochondrial calcium overload or insufficient uptake is aggravating factors of pressure overload heart failure. Thai et al. [138] found that TAC caused damage to mitochondrial Ca^2+^ uptake in mouse cardiomyocytes. Silencing the translocator protein of the outer mitochondrial membrane to restore mitochondrial Ca^2+^ uptake can protect the heart from pathological myocardial hypertrophy and cardiac remodelling caused by pressure overload. Elrod et al. [139] confirmed that Ppif gene deficiency in mice led to a decrease in physical opening of MPTP and an abnormal increase in mitochondrial Ca^2+^, aggravating myocardial hypertrophy and heart failure after pressure overload. MCU anchored in the inner mitochondrial membrane is the most important one-way channel responsible for Ca^2+^ influx into mitochondria [140]. Ca^2+^ is a ubiquitous intracellular signal messenger that participates in many cellular functions, including mitophagy [141]. However, there is still no unified conclusion on how mitochondrial Ca^2+^ triggers and regulates mitophagy in different disease models. In myocardial ischaemia–reperfusion injury model, mitochondrial calcium overload caused by MCU upregulation activated calpain, thus inhibiting OPA1 and mitochondrial fusion, resulting in the inhibition of mitophagy [142]. In vascular smooth muscle cells, MCU-dependent mitochondrial Ca^2+^ uptake promotes mitophagy [143]. MCU is closely related to a variety of mechanisms that mediate mitophagy. The use of MCU inhibitor RU360 in vascular endothelial cells inhibits mitochondrial division by inhibiting DRP1 phosphorylation and oligomers [144]. MCU-dependent mitochondrial Ca^2+^ uptake can also induce mtROS production [145]. The use of RU360 reduces mtROS generation [146]. MPTP opening is a main pathway of physiological mitochondrial Ca^2+^ efflux. MPTP opening plays a decisive role in the activation of Pink1–Parkin-mediated mitophagy [147]. It has been proved that inhibiting MCU will reduce the opening of MPTP, and activating MCU will increase the opening of MPTP [148]. MCU also regulates mitochondrial metabolism by targeting the key enzymes involved in the TCA, through mitochondrial Ca^2+^ uptake [149]. An abnormal TCA cycle will change the biosynthesis of metabolites that have an impact on myocardial hypertrophy. A paper by Ritterhoff et al. [150] showed that remodelling of the TCA cycle promotes the increase of glucose-derived aspartate and promotes myocardial hypertrophy. AKG is an important intermediate of the TCA cycle that regulates a variety of important physiological functions, including cell metabolism and signal transduction. Dietary AKG supplementation inhibits cardiac hypertrophy and fibrosis induced by TAC [48]. An et al. [48] confirmed that TAC causes a decline of Pink1/Parkin, and the use of AKG inhibits this trend and reduces the production of ROS. Current research has established a direct link between MCU, mitophagy, and pressure overload-induced heart failure. In heart failure induced by pressure overload, MCU expression is upregulated, and autophagic flux is blocked. After the use of MCU inhibitors, Parkin and Pink1 are upregulated, mitophagy is enhanced, and cardiac function is improved [151]. These findings suggest that the regulation of mitophagy by MCU is a potential therapeutic target for heart failure induced by pressure overload.

### 4.5. Signalling Pathways Potentially Influencing Mitophagy

AMPK is a key sensor of cellular energy state and is considered a participant in mitophagy. The relationship between AMPK, mitophagy, and pressure overload-induced heart failure has been established. Wang et al. [152] constructed AMPK catalytic *α*2-subunit knockout mice and demonstrated that its absence exacerbates heart failure after TAC by inhibiting mitophagy. Pink1 phosphorylation and Pink1/Parkin-mediated mitophagy were enhanced after AMPK*α*2 overexpression. Several sites on Pink1 can be phosphorylated by AMPK*α*2, but Ser495 residue is considered the optimal site, as Ala mutation reduces mitophagy and induces ROS production there [152]. Phosphorylation of ULK1 is also necessary for mitophagy in the verified case [153]. AMPK can trigger autophagy by activating ULK1 directly or by inhibiting the mTORC1 complex. AMPK mediates the phosphorylation of Ser772 and Ser792 of mTOR binding partner Raptor and is also able to phosphorylate TSC2 upstream of mTOR to jointly inhibit the activity of mTORC1 [154]. Egan et al. [155] identified four AMPK phosphorylated sites in ULK1 (Ser 467, Ser 555, Thr 574, and Ser 637) and confirmed that AMPK or ULK1 knockdown leads to autophagy defects. A recent study determined that GPR39, as an inhibitor of AMPK, increases after TAC to activate mTOR and promotes cardiac hypertrophy [156]. AMPK is also involved in mitochondrial dynamics. DRP1 receptor MFF has two AMPK phosphorylation sites, Ser155 and Ser172, and phosphorylation dysfunction at these two sites prevents DRP1 recruitment to mitochondria [157]. AMPK has also been identified as an upstream signal of OPA1, and inhibition of AMPK results in a decrease in OPA1 expression [51]. Although existing studies have directly linked only part of the mechanism of AMPK regulation of mitophagy to the cardiac phenotype under pressure overload, current results still provide a blueprint for applying the AMPK–mitophagy pathway to the model of pressure overload.

SIRT1 is an NAD^+^-dependent deacetylase that mediates a variety of physiological effects, such as cell metabolism, proliferation, and differentiation [158]. SIRT1 was earlier shown to activate autophagy, but it was also found that there is a significant accumulation of abnormal mitochondria after SIRT1 knockout [159]. Subsequent studies by Huang et al. [160] proved that nicotinamide promoted the increase of [NAD^+^]/[NADH] ratio through the salvage pathway, mediated the enhancement of SIRT1 activity, and thus improved mitophagy. This is favourable evidence that SIRT1 is directly associated with mitophagy. Existing theories are gradually clarifying how SIRT1 is involved in mitophagy through different pathways. Resveratrol is a natural compound with an antiageing effect. It activates SIRT1/SIRT3 to exert cardiac protection through the Pink–Parkin pathway via FOXO3 [161]. Available evidence suggests that SIRT1 plays a protective role in cardiac hypertrophy induced by pressure overload. After SIRT1 knockout, the indexes of myocardial hypertrophy *β*-MHC and ANP increase [162]. SIRT1 can also negatively regulate the mTOR signalling pathway and affect autophagy and mitophagy-mediated mitochondrial clearance [163]. SIRT1 also enables PGC-1*α* deacetylation, which in turn activates the Pink–Parkin pathway [164]. Although the current study is optimistic about the positive role of PGC-1*α* in pressure overload models [165], studies have not established a direct correlation between PGC-1*α*-induced mitophagy and cardiac remodelling induced by pressure overload. Future studies may not rule out the possibility of SIRT1/PGC-1*α*-mediated mitophagy as a therapeutic target for pressure overload.

PTEN is a phosphatase of lipids and proteins that inhibits tumour growth, regulates glucose and lipid metabolism, and adjusts mitochondrial function [166]. PTEN can inhibit the PI3K/AKT pathway and promote autophagy [167]. However, several studies have found that PTEN can inhibit mitophagy. Li et al. [168] confirmed that PTEN restricts mitophagy by inhibiting the TLR4–JNK–BNIP3 pathway. Knockout of PTEN increases the activity of mitophagy by increasing the expression of MFN2 [169]. In the TAC model, inhibition of PTEN degradation led to AKT/mTOR inactivation and AMPK signal activation, thereby ameliorating cardiac hypertrophy and dysfunction caused by pressure overload [170]. The results of Tian et al. [171] showed that in TAC model or ISO induced cardiomyocyte hypertrophy, LKB1IP activates AKT signal transduction by inhibiting the phosphatase activity of PTEN, thereby aggravating pathological cardiac hypertrophy. However, there is no study on the direct connection between PTEN, mitophagy, and pathological cardiac hypertrophy.

The functions of P53 include but are not limited to tumour inhibition, ageing, metabolism regulation, and oxidative stress regulation. Hoshino et al. [172] revealed its role in mitophagy, wherein residues 81–160 of P53 interact with the RING0 region of Parkin and inhibit mitochondrial translocation of Parkin, thereby inhibiting mitophagy. P53 increases significantly one week after TAC [173]. Overexpression of Canopy 2 inhibits the expression of P53 and maintains cardiac structure and function after TAC [173]. Nrf2 is an antioxidant involved in oxidative stress and mitophagy in a variety of disease models. The expression levels of Pink and Parkin are reduced after Nrf2 is knocked out by siRNA [174]. Nrf2 can also be combined with the ARE sequence of P62 to activate the expression of P62. P62 has also been proved to lead to the activation of Nrf2. Their mutual regulation forms a cycle and regulates the homeostasis of mitophagy [175]. Finally, peroxiredoxin 1 was shown to inhibit TAC-induced cardiac remodelling and cardiac dysfunction. Peroxiredoxin 1 increases the expression of Nrf2 after TAC, and knockout of Nrf2 inhibits the protective effect of peroxiredoxin 1 [176].

## 5. Mitophagy and Cardiac Nonmyocytes

Cardiac nonmyocytes actively participate in the development of cardiac hypertrophy under pressure overload. Fibroblasts, vascular endothelial cells, and macrophages are all important in pressure overload-induced cardiac remodelling [177]. Activation of cardiac fibroblasts is a hallmark of cardiac remodelling and fibrosis caused by pressure overload [178]. Cardiac fibroblasts can also promote cardiomyocyte hypertrophy through paracrine communication [177]. Therefore, the control of myocardial fibrotic remodelling is considered a possible target for the treatment of heart failure induced by pressure overload [179]. Activation of cardiac fibroblasts can be regulated by mitophagy. Mitophagy plays a role in tissue fibrosis remodelling [180]. ADAM17, known as disintegrin and metalloproteases, whose knockdown inhibited TGF-*β*1, induced collagen synthesis in cardiac fibroblasts by enhancing mitophagy [181]. However, a study of Zhang et al. [182] suggested that Mir-24-3p reduced myocardial fibrosis by inhibiting mitophagy in mice undergoing TAC surgery. A growing number of studies have reported the complex role of macrophages in cardiac remodelling induced by pressure overload. Huo et al. [128] observed an increase in the infiltration of macrophages in heart tissue at 4 and 8 weeks after TAC. A single-cell sequencing of cells isolated from mouse hearts after TAC showed that macrophage subtype conversion is a key event in the progression of pathological myocardial hypertrophy 2 to 5 weeks after TAC [183]. Macrophages can release cytokines to promote cardiomyocyte hypertrophy and myocardial fibroblast activation [184]. However, cardiac resident macrophages can inhibit myocardial fibrosis and stimulate angiogenesis under pressure overload [185]. Patoli et al. [186] revealed the regulation of mitophagy on macrophage activation; they found that LPS/IFN-*γ*-mediated mitophagy inhibition triggers macrophage activation through ROS. The reduction of adaptive angiogenesis under pressure overload aggravates cardiac dysfunction [187]. Overexpression of SIRT3 in cardiac microvascular endothelial cells enhances Pink/Parkin-mediated mitophagy, reduces the production of ROS, and promotes angiogenesis [188]. The effect of mitophagy on the phenotype of cardiac nonmyocytes reflects the extensive regulation of mitophagy in pathological changes of the heart under pressure overload and further clarifies the significant impact mitophagy will have in the identification of new therapeutic targets for cardiac remodelling and heart failure under pressure overload.

## 6. Active Compounds with the Potential to Intervene in the Effects of Pressure Overload on the Heart by Regulating Mitophagy

There is as yet no general clinical consensus on intervening in mitophagy under pressure overload. However, the current research provides promising pathways and new starting points for the treatment of heart injury caused by pressure overload, covering as it does multiple aspects of mitophagy. The latest view takes a short-term high-fat diet as a measure to inhibit cardiac hypertrophy after TAC. A short-term high-fat diet enhances the utilisation of fatty acids in the myocardium and enhances mitophagy by upregulating Parkin, which provides novel evidence for the effect of diet on mitophagy [189]. The researchers in the cited study also found that a long-term high-fat diet did not enhance mitophagy and even caused lipotoxic damage to the myocardium. Therefore, it is indicated that the regulation of mitophagy by diet requires precise timing and careful use [189]. There is broad consensus that statins improve the outcomes of heart failure. In the case of pressure overload, the combination of simvastatin and losartan reduces cardiac remodelling. In the detection of Parkin and observation of ultrastructure by transmission electron microscope, mitophagy was considered involved in the protective effect of simvastatin [190]. A variety of natural herbal active compounds have also been shown to regulate mitophagy in the pressure overload model. Berberine is extracted from Coptis Chinensis, and its protective effect on the heart has been confirmed in recent years [191]. Abudureyimu et al. [113] found that Berberine alleviates the inhibition of mitophagy after TAC through the Pink–Parkin pathway, reduces the accumulation of swelling and damaged mitochondria, and reduces ROS levels. Inhibition of the mTOR pathway by Berberine has also been demonstrated in vivo and in vitro in response to cardiac remodelling induced by TAC [191]. Baicalein can be combined with FOXO3a, which plays a protective role in the pressure overload model, and increases the mRNA and protein levels of FUNDC1 after TAC [192].

## 7. Conclusion and Future Perspectives

In pressure overload-induced cardiac remodelling, mitochondrial damage exerts negative effects by interfering with normal energy metabolism and mediating oxidative stress and mtDNA imbalance. Many studies support that mitophagy is a cell-initiated protective mechanism to protect the heart from various effects of mitochondrial damage. Mitophagy not only plays a role in the TAC model but also plays a protective role in Ang II-induced myocardial injury and hypertensive cardiac remodelling [188, 193]. However, the regulation of mitochondrial dynamics, mitophagy pathways, and related signal transduction in pressure overload must be the comprehensively investigated. The roles of genes, drugs, and active molecules in mitophagy indicate many meaningful targets for ameliorating the adverse effects of pressure overload. This paper has also summarised the protective effects of conventional clinical drugs on the heart under stress overload by regulating mitophagy. However, a limitation is that most studies have been conducted at cytological and zoological levels, and few studies have been used for clinical validation. Precise targets and drugs for manipulating mitophagy need to be developed to treat cardiac dysfunction caused by pressure overload.

## Figures and Tables

**Figure 1:** Overview of mitophagy. Mitophagy is a selective autophagy that maintains physiological functions by selectively degradation of damaged or dysfunctional mitochondria. During mitophagy, the damaged mitochondria are labeled and surrounded by vesicles which stretch to form autophagosome. Lastly, autophagosomes fuse with lysosomes to form autophagolysosomes, where hydrolases degrade the sequestered materials and released the degraded products into cytoplasm.

**Figure 2:** Mitochondria-related damage and potential role of mitophagy in pressure overload model. More mitochondrial cristae disorders, decreased cristae density, and mitochondrial swelling appear after pressure overloaded. Mitochondrial respiration is impaired. Oxidative stress is an important mediator in the mechanism of pathological cardiac remodelling. Under pressure overload, a variety of mechanisms regulate the increase of ROS and RNS. Under pressure overload, ROS and a variety of upstream signals also lead to mtDNA damage, resulting in pathological cardiac remodelling. mtDNA damage and ROS activate mitophagy through a variety of mechanisms. Mitophagy inhibits the adverse effects of ROS and mtDNA.

**Figure 3:** Mitochondrial dynamics in pressure overload model. In the pressure overload model, MFN2 was downregulated. After TAC, Mir-17-5p and Mir-106a inhibit MFN2 and cause cardiac hypertrophy. In OPA1+/- mice, TAC results in more severe cardiac remodelling and cardiac dysfunction. Increased expression of OPA1 by upregulating YME1L or TNFR2 protects hearts from pressure overload. The decreased level phosphorylation at s616 of DRP1 accompanies a decrease in mitophagy. Knockout of DRP1 aggravates mitochondrial dysfunction, cardiac hypertrophy, and cardiac dysfunction caused by pressure overload. STAT1 promotes mitochondrial division through UCP2/P-DRP1 pathway to resist TAC-induced myocardial hypertrophy. However, the use of DRP1 inhibitor Mdivi-1 improves cardiac dysfunction and cardiac remodelling after TAC.

## Data Availability

The figures used to support the findings of this review were included within the article.

## Abbreviations

mtDNA: Mitochondrial DNA
TAC: Transverse aortic constriction
ETC: Electron transport chain
AMS: Allyl methyl sulfide
ROS: Reactive oxygen species
RNS: Reactive nitrogen species
NOXs: NADPH oxidases
BH4: Tetrahydrobiopterin
NOS: Nitric oxide synthase
Ffar4: Free fatty acid receptor 4
JMJD: JmjC domain-containing
Pol *γ*: DNA polymerase *γ*
NDUFS1: NADH-ubiquinone oxidoreductase 75 kDa subunit
TGF-*β*1: Transforming growth factor *β*1
TIGAR: TP53-induced glycolysis and apoptosis regulator
BNIP3: BCL2 and adenovirus E1B 19 kDa-interacting protein 3
NIX: BNIP3-like
ATG: Autophagy-related proteins
FOXO3: Factor forkhead box O-3
Nrf2: Nuclear factor erythroid 2-related factor 2
ATAD3B: AAA-domain-containing protein 3B
OPA1: Optic atrophy 1
MFN: Mitochondrial fusion protein
IMS: Intermembrane space
DRP1: Dynein-related protein 1
FIS1: Mitochondrial fission protein 1
MFF: Mitochondrial fission factor
MID: Mitochondrial dynamics proteins
MEF: Murine embryonic fibroblasts
CCCP: Carbonyl cyanide m-chlorophenylhydrazone
STX: Syntaxin
TNFR2: TNF*α* receptor 2
MTS: Mitochondrial targeting sequence
Tom: Mitochondrial outer membrane transporter
TIM: Mitochondrial inner membrane transporter
MOM: Mitochondrial outer membrane
VDAC1: Voltage-dependent anion channel 1
Miro: Rho GTPase of mitochondrial
RAGE: Receptor for advanced glycation end products
MAM: Mitochondria-associated membrane
IP3R2: Inositol 1,4,5-trisphosphate type 2 receptor
FUNDC1: FUN14 domain-containing 1
*α*-LA: Alpha-lipoic acid
MPTP: Mitochondrial permeability transition pore
MCU: Mitochondrial calcium uniporter
mtROS: Mitochondrial ROS
TCA cycle: Tricarboxylic acid cycle
AKG: *α*-Ketoglutarate
mTOR: Mechanistic target of rapamycin
ULK1: Unc-51 like autophagy activating kinase 1
SIRT1: Sirtuin1
PGC-1*α*: Peroxisome proliferator-activated receptor gamma coactivator 1 alpha
PTEN: Phosphatase and tensin homolog deleted on chromosome 10

## References

[1] Houser S. R., Margulies K. B., Murphy A. M. (2012). Animal models of heart failure. *Circulation Research*.

[2] Shimizu I., Minamino T. (2016). Physiological and pathological cardiac hypertrophy. *Journal of Molecular and Cellular Cardiology*.

[3] Zeng D., Chen H., Jiang C. L., Wu J. (2017). Usefulness of three-dimensional spherical index to assess different types of left ventricular remodeling: a meta-analysis. *Medicine*.

[4] Mesías A. C., Garg N. J., Zago M. P. (2019). Redox balance keepers and possible cell functions managed by redox homeostasis in trypanosoma cruzi. *Frontiers in Cellular and Infection Microbiology*.

[5] Aravamudan B., Thompson M. A., Pabelick C. M., Prakash Y. S. (2013). Mitochondria in lung diseases. *Expert Review of Respiratory Medicine*.

[6] Friedman J. R., Nunnari J. (2014). Mitochondrial form and function. *Nature*.

[7] Shu H., Hang W., Peng Y. (2021). Trimetazidine attenuates heart failure by improving myocardial metabolism via AMPK. *Frontiers in Pharmacology*.

[8] Shen C., Wang C., Fan F. (2015). Acetaldehyde dehydrogenase 2 (ALDH2) deficiency exacerbates pressure overload- induced cardiac dysfunction by inhibiting Beclin-1 dependent autophagy pathway. *Biochimica et Biophysica Acta*.

[9] Liang K. X., Kristiansen C. K., Mostafavi S. (2020). Disease-specific phenotypes in iPSC-derived neural stem cells with POLG mutations. *EMBO Molecular Medicine*.

[10] Schwarzer M., Osterholt M., Lunkenbein A., Schrepper A., Amorim P., Doenst T. (2014). Mitochondrial reactive oxygen species production and respiratory complex activity in rats with pressure overload-induced heart failure. *The Journal of Physiology*.

[11] Bugger H., Schwarzer M., Chen D. (2010). Proteomic remodelling of mitochondrial oxidative pathways in pressure overload-induced heart failure. *Cardiovascular Research*.

[12] Jüllig M., Hickey A. J., Chai C. C. (2008). Is the failing heart out of fuel or a worn engine running rich? A study of mitochondria in old spontaneously hypertensive rats. *Proteomics*.

[13] Griffiths E. R., Friehs I., Scherr E., Poutias D., McGowan F. X., del Nido P. J. (2010). Electron transport chain dysfunction in neonatal pressure-overload hypertrophy precedes cardiomyocyte apoptosis independent of oxidative stress. *The Journal of Thoracic and Cardiovascular Surgery*.

[14] Dai D. F., Hsieh E. J., Liu Y. (2012). Mitochondrial proteome remodelling in pressure overload-induced heart failure: the role of mitochondrial oxidative stress. *Cardiovascular Research*.

[15] Ribeiro Junior R. F., Dabkowski E. R., Shekar K. C., O´Connell K. A., Hecker P. A., Murphy M. P. (2018). MitoQ improves mitochondrial dysfunction in heart failure induced by pressure overload. *Free Radical Biology & Medicine*.

[16] Mohammed S. A., Paramesha B., Meghwani H., Kumar Reddy M. P., Arava S. K., Banerjee S. K. (2021). Allyl methyl sulfide preserved pressure overload-induced heart failure via modulation of mitochondrial function. *Biomedicine & Pharmacotherapy*.

[17] Garza-Lombó C., Pappa A., Panayiotidis M. I., Franco R. (2020). Redox homeostasis, oxidative stress and mitophagy. *Mitochondrion*.

[18] Prasad K., Gupta J. B., Kalra J., Lee P., Mantha S. V., Bharadwaj B. (1996). Oxidative stress as a mechanism of cardiac failure in chronic volume overload in canine model. *Journal of Molecular and Cellular Cardiology*.

[19] Eiki T., Kass D. A. (2007). Role of oxidative stress in cardiac hypertrophy and remodeling. *Hypertension*.

[20] Tsutsui H., Kinugawa S., Matsushima S. (2011). Oxidative stress and heart failure. *American Journal of Physiology. Heart and Circulatory Physiology*.

[21] Kussmaul L., Hirst J. (2006). The mechanism of superoxide production by NADH:ubiquinone oxidoreductase (complex I) from bovine heart mitochondria. *Proceedings of the National Academy of Sciences of the United States of America*.

[22] Muller F. L., Liu Y., Van Remmen H. (2004). Complex III releases superoxide to both sides of the inner mitochondrial membrane∗. *The Journal of Biological Chemistry*.

[23] Bedard K., Krause K. H. (2007). The NOX family of ROS-generating NADPH oxidases: physiology and pathophysiology. *Physiological Reviews*.

[24] Kuroda J., Ago T., Matsushima S., Zhai P., Schneider M. D., Sadoshima J. (2010). NADPH oxidase 4 (Nox4) is a major source of oxidative stress in the failing heart. *Proceedings of the National Academy of Sciences of the United States of America*.

[25] Shimizu S., Ishibashi M., Kumagai S. (2013). Decreased cardiac mitochondrial tetrahydrobiopterin in a rat model of pressure overload. *International Journal of Molecular Medicine*.

[26] Fukai T., Ushio-Fukai M. (2011). Superoxide dismutases: role in redox signaling, vascular function, and diseases. *Antioxidants & Redox Signaling*.

[27] Filipovic M. R., Koppenol W. H. (2019). The Haber-Weiss reaction - the latest revival. *Free Radical Biology & Medicine*.

[28] Brown G. C., Borutaite V. (2004). Inhibition of mitochondrial respiratory complex I by nitric oxide, peroxynitrite and S-nitrosothiols. *Biochimica et Biophysica Acta*.

[29] Borbély A., Tóth A., Edes I. (2005). Peroxynitrite-induced alpha-actinin nitration and contractile alterations in isolated human myocardial cells. *Cardiovascular Research*.

[30] Zou M. H., Shi C., Cohen R. A. (2002). Oxidation of the zinc-thiolate complex and uncoupling of endothelial nitric oxide synthase by peroxynitrite. *The Journal of Clinical Investigation*.

[31] Takimoto E., Champion H. C., Li M. (2005). Oxidant stress from nitric oxide synthase-3 uncoupling stimulates cardiac pathologic remodeling from chronic pressure load. *The Journal of Clinical Investigation*.

[32] Moens A. L., Leyton-Mange J. S., Niu X. (2009). Adverse ventricular remodeling and exacerbated NOS uncoupling from pressure- overload in mice lacking the *β*3-adrenoreceptor. *Journal of Molecular and Cellular Cardiology*.

[33] Murphy K. A., Harsch B. A., Healy C. L. (2022). Free fatty acid receptor 4 responds to endogenous fatty acids to protect the heart from pressure overload. *Cardiovascular Research*.

[34] Zang R., Tan Q., Zeng F., Wang D., Yu S., Wang Q. (2020). JMJD1A represses the development of cardiomyocyte hypertrophy by regulating the expression of catalase. *BioMed Research International*.

[35] Mao K., Breen P., Ruvkun G. (2020). Mitochondrial dysfunction induces RNA interference in C. elegans through a pathway homologous to the mammalian RIG-I antiviral response. *PLoS Biology*.

[36] Yue R., Xia X., Jiang J. (2015). Mitochondrial DNA oxidative damage contributes to cardiomyocyte ischemia/reperfusion-injury in rats: cardioprotective role of lycopene. *Journal of Cellular Physiology*.

[37] Marín-García J. (2016). Mitochondrial DNA repair: a novel therapeutic target for heart failure. *Heart Failure Reviews*.

[38] Anderson A. P., Luo X., Russell W., Yin Y. W. (2020). Oxidative damage diminishes mitochondrial DNA polymerase replication fidelity. *Nucleic Acids Research*.

[39] Shokolenko I., Venediktova N., Bochkareva A., Wilson G. L., Alexeyev M. F. (2009). Oxidative stress induces degradation of mitochondrial DNA. *Nucleic Acids Research*.

[40] Zou R., Tao J., Qiu J. (2021). Ndufs1 deficiency aggravates the mitochondrial membrane potential dysfunction in pressure overload-induced myocardial hypertrophy. *Oxidative Medicine and Cellular Longevity*.

[41] Sen D., Nandakumar D., Tang G. Q., Patel S. S. (2012). Human mitochondrial DNA helicase TWINKLE is both an unwinding and annealing helicase. *Journal of Biological Chemistry*.

[42] Tanaka A., Ide T., Fujino T. (2013). The overexpression of Twinkle helicase ameliorates the progression of cardiac fibrosis and heart failure in pressure overload model in mice. *PLoS One*.

[43] Sharma B., Chaube U., Patel B. M. (2019). Beneficial effect of silymarin in pressure overload induced experimental cardiac hypertrophy. *Cardiovascular Toxicology*.

[44] Li L., Tan J., Miao Y., Lei P., Zhang Q. (2015). ROS and autophagy: interactions and molecular regulatory mechanisms. *Cellular and Molecular Neurobiology*.

[45] Xiao B., Deng X., Lim G. G. (2017). Superoxide drives progression of Parkin/PINK1-dependent mitophagy following translocation of Parkin to mitochondria. *Cell death & disease*.

[46] Oh C. K., Sultan A., Platzer J. (2017). S-Nitrosylation of PINK1 attenuates PINK1/Parkin-dependent mitophagy in hiPSC-based Parkinson’s disease models. *Cell Reports*.

[47] Ozawa K., Komatsubara A. T., Nishimura Y. (2013). S-Nitrosylation regulates mitochondrial quality control via activation of parkin. *Scientific Reports*.

[48] An D., Zeng Q., Zhang P. (2021). Alpha-ketoglutarate ameliorates pressure overload-induced chronic cardiac dysfunction in mice. *Redox Biology*.

[49] Kandul N. P., Zhang T., Hay B. A., Guo M. (2016). Selective removal of deletion-bearing mitochondrial DNA in heteroplasmic drosophila. *Nature Communications*.

[50] Shu L., Hu C., Xu M. (2021). ATAD3B is a mitophagy receptor mediating clearance of oxidative stress-induced damaged mitochondrial DNA. *The EMBO Journal*.

[51] Zhang Y., Wang Y., Xu J. (2019). Melatonin attenuates myocardial ischemia-reperfusion injury via improving mitochondrial fusion/mitophagy and activating the AMPK-OPA1 signaling pathways. *Journal of Pineal Research*.

[52] Jin Q., Li R., Hu N. (2018). DUSP1 alleviates cardiac ischemia/reperfusion injury by suppressing the Mff- required mitochondrial fission and Bnip3-related mitophagy via the JNK pathways. *Redox Biology*.

[53] Youle R. J., van der Bliek A. M. (2012). Mitochondrial fission, fusion, and stress. *Science*.

[54] Sciarretta S., Maejima Y., Zablocki D., Sadoshima J. (2018). The role of autophagy in the heart. *Annual Review of Physiology*.

[55] Yu R., Lendahl U., Nistér M., Zhao J. (2020). Regulation of mammalian mitochondrial dynamics: opportunities and challenges. *Frontiers in endocrinology*.

[56] Mattie S., Riemer J., Wideman J. G., McBride H. M. (2018). A new mitofusin topology places the redox-regulated C terminus in the mitochondrial intermembrane space. *The Journal of Cell Biology*.

[57] Cao Y. L., Meng S., Chen Y. (2017). MFN1 structures reveal nucleotide-triggered dimerization critical for mitochondrial fusion. *Nature*.

[58] Chen H., Detmer S. A., Ewald A. J., Griffin E. E., Fraser S. E., Chan D. C. (2003). Mitofusins Mfn1 and Mfn2 coordinately regulate mitochondrial fusion and are essential for embryonic development. *The Journal of Cell Biology*.

[59] Song Z., Ghochani M., McCaffery J. M., Frey T. G., Chan D. C. (2009). Mitofusins and OPA1 mediate sequential steps in mitochondrial membrane fusion. *Molecular Biology of the Cell*.

[60] Song Z., Chen H., Fiket M., Alexander C., Chan D. C. (2007). OPA1 processing controls mitochondrial fusion and is regulated by mRNA splicing, membrane potential, and Yme1L. *The Journal of Cell Biology*.

[61] Zhang D., Zhang Y., Ma J. (2020). Cryo-EM structures of S-OPA1 reveal its interactions with membrane and changes upon nucleotide binding. *eLife*.

[62] Ge Y., Shi X., Boopathy S., McDonald J., Smith A. W., Chao L. H. (2020). Two forms of Opa1 cooperate to complete fusion of the mitochondrial inner-membrane. *eLife*.

[63] Ingerman E., Perkins E. M., Marino M. (2005). Dnm1 forms spirals that are structurally tailored to fit mitochondria. *The Journal of Cell Biology*.

[64] Otera H., Ishihara N., Mihara K. (2013). New insights into the function and regulation of mitochondrial fission. *Biochimica et Biophysica Acta*.

[65] Otera H., Wang C., Cleland M. M. (2010). Mff is an essential factor for mitochondrial recruitment of Drp1 during mitochondrial fission in mammalian cells. *The Journal of Cell Biology*.

[66] Losón O. C., Song Z., Chen H., Chan D. C. (2013). Fis1, Mff, MiD49, and MiD51 mediate Drp1 recruitment in mitochondrial fission. *Molecular Biology of the Cell*.

[67] Liu T., Yu R., Jin S. B. (2013). The mitochondrial elongation factors MIEF1 and MIEF2 exert partially distinct functions in mitochondrial dynamics. *Experimental Cell Research*.

[68] Zhao J., Liu T., Jin S. (2011). Human MIEF1 recruits Drp1 to mitochondrial outer membranes and promotes mitochondrial fusion rather than fission. *The EMBO Journal*.

[69] Lee Y. J., Jeong S. Y., Karbowski M., Smith C. L., Youle R. J. (2004). Roles of the mammalian mitochondrial fission and fusion mediators Fis1, Drp1, and Opa1 in apoptosis. *Molecular Biology of the Cell*.

[70] Twig G., Elorza A., Molina A. J. (2008). Fission and selective fusion govern mitochondrial segregation and elimination by autophagy. *The EMBO Journal*.

[71] Song M., Mihara K., Chen Y., Scorrano L., Dorn G. W. (2015). Mitochondrial fission and fusion factors reciprocally orchestrate mitophagic culling in mouse hearts and cultured fibroblasts. *Cell Metabolism*.

[72] Chen Y., Dorn G. W. (2013). PINK1-phosphorylated mitofusin 2 is a Parkin receptor for culling damaged mitochondria. *Science*.

[73] Zhao T., Huang X., Han L. (2012). Central Role of Mitofusin 2 in Autophagosome-Lysosome Fusion in Cardiomyocytes∗. *The Journal of Biological Chemistry*.

[74] de Brito O. M., Scorrano L. (2008). Mitofusin 2 tethers endoplasmic reticulum to mitochondria. *Nature*.

[75] Liao C., Ashley N., Diot A. (2017). Dysregulated mitophagy and mitochondrial organization in optic atrophy due to OPA1 mutations. *Neurology*.

[76] Xin T., Lu C. (2020). Irisin activates Opa1-induced mitophagy to protect cardiomyocytes against apoptosis following myocardial infarction. *Aging*.

[77] Lee Y., Lee H. Y., Hanna R. A., Gustafsson Å. B. (2011). Mitochondrial autophagy by Bnip3 involves Drp1-mediated mitochondrial fission and recruitment of Parkin in cardiac myocytes. *American Journal of Physiology. Heart and Circulatory Physiology*.

[78] Ikeda Y., Shirakabe A., Maejima Y. (2015). Endogenous Drp1 mediates mitochondrial autophagy and protects the heart against energy stress. *Circulation Research*.

[79] Mao K., Wang K., Liu X., Klionsky D. J. (2013). The scaffold protein Atg11 recruits fission machinery to drive selective mitochondria degradation by autophagy. *Developmental Cell*.

[80] Yamashita S. I., Kanki T. (2017). How autophagy eats large mitochondria: autophagosome formation coupled with mitochondrial fragmentation. *Autophagy*.

[81] Burman J. L., Pickles S., Wang C. (2017). Mitochondrial fission facilitates the selective mitophagy of protein aggregates. *The Journal of Cell Biology*.

[82] Gao J., Qin S., Jiang C. (2015). Parkin-induced ubiquitination of Mff promotes its association with p62/SQSTM1 during mitochondrial depolarization. *Acta Biochimica et Biophysica Sinica*.

[83] Xian H., Liou Y. C. (2019). Loss of MIEF1/MiD51 confers susceptibility to BAX-mediated cell death and PINK1-PRKN-dependent mitophagy. *Autophagy*.

[84] Gomes L. C., Scorrano L. (2008). High levels of Fis1, a pro-fission mitochondrial protein, trigger autophagy. *Biochimica et Biophysica Acta*.

[85] Yamano K., Fogel A. I., Wang C., van der Bliek A. M., Youle R. J. (2014). Mitochondrial Rab GAPs govern autophagosome biogenesis during mitophagy. *eLife*.

[86] Arasaki K., Shimizu H., Mogari H. (2015). A role for the ancient SNARE syntaxin 17 in regulating mitochondrial division. *Developmental Cell*.

[87] Xian H., Yang Q., Xiao L., Shen H. M., Liou Y. C. (2019). STX17 dynamically regulated by Fis1 induces mitophagy via hierarchical macroautophagic mechanism. *Nature Communications*.

[88] Alavi M. V., Fuhrmann N., Nguyen H. P. (2009). Subtle neurological and metabolic abnormalities in an _Opa1_ mouse model of autosomal dominant optic atrophy. *Experimental Neurology*.

[89] Zaha K., Matsumoto H., Itoh M. (2016). DNM1L-related encephalopathy in infancy with Leigh syndrome-like phenotype and suppression-burst. *Clinical Genetics*.

[90] Fang L., Moore X. L., Gao X. M., Dart A. M., Lim Y. L., du X. J. (2007). Down-regulation of mitofusin-2 expression in cardiac hypertrophy in vitro and in vivo. *Life Sciences*.

[91] Xiong W., Ma Z., An D. (2019). Mitofusin 2 participates in Mitophagy and mitochondrial fusion against angiotensin II-induced cardiomyocyte injury. *Frontiers in Physiology*.

[92] Xu X., Su Y. L., Shi J. Y., Lu Q., Chen C. (2021). MicroRNA-17-5p promotes cardiac hypertrophy by targeting Mfn2 to inhibit autophagy. *Cardiovascular Toxicology*.

[93] Guan X., Wang L., Liu Z. (2016). miR-106a promotes cardiac hypertrophy by targeting mitofusin 2. *Journal of Molecular and Cellular Cardiology*.

[94] Piquereau J., Caffin F., Novotova M. (2012). Down-regulation of OPA1 alters mouse mitochondrial morphology, PTP function, and cardiac adaptation to pressure overload. *Cardiovascular Research*.

[95] Guo Y., Wang Z., Qin X. (2018). Enhancing fatty acid utilization ameliorates mitochondrial fragmentation and cardiac dysfunction via rebalancing optic atrophy 1 processing in the failing heart. *Cardiovascular Research*.

[96] Nan J., Hu H., Sun Y. (2017). TNFR2 stimulation promotes mitochondrial fusion via Stat3- and NF-kB-dependent activation of OPA1 expression. *Circulation Research*.

[97] Shirakabe A., Zhai P., Ikeda Y. (2016). Drp1-dependent mitochondrial autophagy plays a protective role against pressure overload-induced mitochondrial dysfunction and heart failure. *Circulation*.

[98] Ma M., Chen W., Hua Y., Jia H., Song Y., Wang Y. (2021). Aerobic exercise ameliorates cardiac hypertrophy by regulating mitochondrial quality control and endoplasmic reticulum stress through M2AChR. *Journal of Cellular Physiology*.

[99] Givvimani S., Munjal C., Tyagi N., Sen U., Metreveli N., Tyagi S. C. (2012). Mitochondrial division/mitophagy inhibitor (Mdivi) ameliorates pressure overload induced heart failure. *PLoS One*.

[100] Valente E. M., Abou-Sleiman P. M., Caputo V. (2004). Hereditary early-onset Parkinson's disease caused by mutations in PINK1. *Science*.

[101] Sekine S., Youle R. J. (2018). PINK1 import regulation; a fine system to convey mitochondrial stress to the cytosol. *BMC Biology*.

[102] Greene A. W., Grenier K., Aguileta M. A. (2012). Mitochondrial processing peptidase regulates PINK1 processing, import and Parkin recruitment. *EMBO Reports*.

[103] Deas E., Plun-Favreau H., Gandhi S. (2011). PINK1 cleavage at position A103 by the mitochondrial protease PARL. *Human Molecular Genetics*.

[104] Trempe J. F., Sauvé V., Grenier K. (2013). Structure of parkin reveals mechanisms for ubiquitin ligase activation. *Science*.

[105] Riley B. E., Lougheed J. C., Callaway K. (2013). Structure and function of Parkin E3 ubiquitin ligase reveals aspects of RING and HECT ligases. *Nature Communications*.

[106] Meng Y., Qiao H., Ding J. (2020). Effect of Parkin on methamphetamine-induced *α*-synuclein degradation dysfunction in vitro and in vivo. *Brain and Behavior: A Cognitive Neuroscience Perspective*.

[107] Narendra D. P., Jin S. M., Tanaka A. (2010). PINK1 is selectively stabilized on impaired mitochondria to activate Parkin. *PLoS Biology*.

[108] Okatsu K., Oka T., Iguchi M. (2012). PINK1 autophosphorylation upon membrane potential dissipation is essential for Parkin recruitment to damaged mitochondria. *Nature Communications*.

[109] Parikh S. M., Yang Y., He L., Tang C., Zhan M., Dong Z. (2015). Mitochondrial function and disturbances in the septic kidney. *Seminars in Nephrology*.

[110] Kondapalli C., Kazlauskaite A., Zhang N. (2012). PINK1 is activated by mitochondrial membrane potential depolarization and stimulates Parkin E3 ligase activity by phosphorylating serine 65. *Open Biology*.

[111] Schmidt M. F., Gan Z. Y., Komander D., Dewson G. (2021). Ubiquitin signalling in neurodegeneration: mechanisms and therapeutic opportunities. *Cell Death and Differentiation*.

[112] Lazarou M., Sliter D. A., Kane L. A. (2015). The ubiquitin kinase PINK1 recruits autophagy receptors to induce mitophagy. *Nature*.

[113] Abudureyimu M., Yu W., Cao R. Y., Zhang Y., Liu H., Zheng H. (2020). Berberine promotes cardiac function by upregulating PINK1/Parkin-mediated Mitophagy in heart failure. *Frontiers in Physiology*.

[114] Cao Y., Xu C., Ye J. (2019). Miro2 regulates inter-mitochondrial communication in the heart and protects against TAC-induced cardiac dysfunction. *Circulation Research*.

[115] Zhang J., Ney P. A. (2009). Role of BNIP3 and NIX in cell death, autophagy, and mitophagy. *Cell Death and Differentiation*.

[116] Glover L. (2020). mSphere of influence: expanding the CRISPR sphere with single-locus proteomics. *mSphere*.

[117] Sulistijo E. S., MacKenzie K. R. (2006). Sequence dependence of BNIP3 transmembrane domain dimerization implicates side-chain hydrogen bonding and a tandem GxxxG motif in specific helix-helix interactions. *Journal of Molecular Biology*.

[118] Hanna R. A., Quinsay M. N., Orogo A. M., Giang K., Rikka S., Gustafsson Å. B. (2012). Microtubule-associated Protein 1 Light Chain 3 (LC3) Interacts with Bnip3 Protein to Selectively Remove Endoplasmic Reticulum and Mitochondria via Autophagy∗. *The Journal of Biological Chemistry*.

[119] Zhu Y., Massen S., Terenzio M. (2013). Modulation of Serines 17 and 24 in the LC3-interacting Region of Bnip3 Determines Pro-survival Mitophagy _versus_ Apoptosis∗. *The Journal of Biological Chemistry*.

[120] Schweers R. L., Zhang J., Randall M. S. (2007). NIX is required for programmed mitochondrial clearance during reticulocyte maturation. *Proceedings of the National Academy of Sciences of the United States of America*.

[121] Sandoval H., Thiagarajan P., Dasgupta S. K. (2008). Essential role for nix in autophagic maturation of erythroid cells. *Nature*.

[122] Yuan Y., Zheng Y., Zhang X. (2017). BNIP3L/NIX-mediated mitophagy protects against ischemic brain injury independent of PARK2. *Autophagy*.

[123] Novak I., Kirkin V., McEwan D. G. (2010). Nix is a selective autophagy receptor for mitochondrial clearance. *EMBO Reports*.

[124] Marinković M., Šprung M., Novak I. (2021). Dimerization of mitophagy receptor BNIP3L/NIX is essential for recruitment of autophagic machinery. *Autophagy*.

[125] Zhang T., Xue L., Li L. (2016). BNIP3 Protein Suppresses PINK1 Kinase Proteolytic Cleavage to Promote Mitophagy∗. *The Journal of Biological Chemistry*.

[126] Chaanine A. H., Jeong D., Liang L. (2012). JNK modulates FOXO3a for the expression of the mitochondrial death and mitophagy marker BNIP3 in pathological hypertrophy and in heart failure. *Cell Death & Disease*.

[127] Gao W., Zhou Z., Liang B. (2018). Inhibiting receptor of advanced glycation end products attenuates pressure overload-induced cardiac dysfunction by preventing excessive autophagy. *Frontiers in Physiology*.

[128] Huo S., Shi W., Ma H. (2021). Alleviation of inflammation and oxidative stress in pressure overload-induced cardiac remodeling and heart failure via IL-6/STAT3 inhibition by Raloxifene. *Oxidative Medicine and Cellular Longevity*.

[129] Liu W., Wang X., Gong J. (2014). The stress-related hormone norepinephrine induced upregulation of nix, contributing to ECM protein expression. *Cell Stress & Chaperones*.

[130] Weng Y. J., Kuo W. W., Kuo C. H. (2010). BNIP3 induces IL6 and calcineurin/NFAT3 hypertrophic-related pathways in H9c2 cardiomyoblast cells. *Molecular and Cellular Biochemistry*.

[131] Liu L., Feng D., Chen G. (2012). Mitochondrial outer-membrane protein FUNDC1 mediates hypoxia-induced mitophagy in mammalian cells. *Nature Cell Biology*.

[132] Lv M., Wang C., Li F. (2017). Structural insights into the recognition of phosphorylated FUNDC1 by LC3B in mitophagy. *Protein & Cell*.

[133] Park S. Y., Koh H. C. (2020). FUNDC1 regulates receptor-mediated mitophagy independently of the PINK1/Parkin-dependent pathway in rotenone-treated SH-SY5Y cells. *Food and Chemical Toxicology*.

[134] Wu S., Lu Q., Wang Q. (2017). Binding of FUN14 domain containing 1 with inositol 1,4,5-trisphosphate receptor in mitochondria-associated endoplasmic reticulum membranes maintains mitochondrial dynamics and function in hearts in vivo. *Circulation*.

[135] Wu W., Lin C., Wu K. (2016). FUNDC1 regulates mitochondrial dynamics at the ER-mitochondrial contact site under hypoxic conditions. *The EMBO Journal*.

[136] Zhang L., Zou J., Chai E., Qi Y., Zhang Y. (2014). Alpha-lipoic acid attenuates cardiac hypertrophy via downregulation of PARP-2 and subsequent activation of SIRT-1. *European Journal of Pharmacology*.

[137] Li W., Yin L., Sun X. (2020). Alpha-lipoic acid protects against pressure overload-induced heart failure via ALDH2-dependent Nrf1-FUNDC1 signaling. *Cell Death & Disease*.

[138] Thai P. N., Daugherty D. J., Frederich B. J. (2018). Cardiac-specific conditional knockout of the 18-kDa mitochondrial translocator protein protects from pressure overload induced heart failure. *Scientific Reports*.

[139] Elrod J. W., Wong R., Mishra S. (2010). Cyclophilin D controls mitochondrial pore-dependent ca(2+) exchange, metabolic flexibility, and propensity for heart failure in mice. *The Journal of Clinical Investigation*.

[140] Xie L., Zhou T., Xie Y., Bode A. M., Cao Y. (2021). Mitochondria-shaping proteins and chemotherapy. *Frontiers in Oncology*.

[141] Gastaldello A., Callaghan H., Gami P., Campanella M. (2010). Ca 2+ -dependent autophagy is enhanced by the pharmacological agent PK11195. *Autophagy*.

[142] Guan L., Che Z., Meng X. (2019). MCU Up-regulation contributes to myocardial ischemia-reperfusion Injury through calpain/OPA-1–mediated mitochondrial fusion/mitophagy Inhibition. *Journal of Cellular and Molecular Medicine*.

[143] Chen Z., Zhou Q., Chen J. (2022). MCU-dependent mitochondrial calcium uptake-induced mitophagy contributes to apelin-13-stimulated VSMCs proliferation. *Vascular Pharmacology*.

[144] Li S., Chen J., Liu M. (2021). Protective effect of HINT2 on mitochondrial function via repressing MCU complex activation attenuates cardiac microvascular ischemia-reperfusion injury. *Basic Research in Cardiology*.

[145] Gu L., Larson Casey J. L., Andrabi S. A. (2019). Mitochondrial calcium uniporter regulates PGC-1*α* expression to mediate metabolic reprogramming in pulmonary fibrosis. *Redox Biology*.

[146] Sripetchwandee J., KenKnight S. B., Sanit J., Chattipakorn S., Chattipakorn N. (2014). Blockade of mitochondrial calcium uniporter prevents cardiac mitochondrial dysfunction caused by iron overload. *Acta Physiologica*.

[147] Zhou H., Zhang Y., Hu S. (2017). Melatonin protects cardiac microvasculature against ischemia/reperfusion injury via suppression of mitochondrial fission-VDAC1-HK2-mPTP-mitophagy axis. *Journal of Pineal Research*.

[148] Yu N., Wang S., Wang P. (2012). The calcium uniporter regulates the permeability transition pore in isolated cortical mitochondria. *Neural Regeneration Research*.

[149] Dong H., Zhao B., Chen J. (2022). Mitochondrial calcium uniporter promotes phagocytosis-dependent activation of the NLRP3 inflammasome. *Proceedings of the National Academy of Sciences of the United States of America*.

[150] Ritterhoff J., Young S., Villet O. (2020). Metabolic remodeling promotes cardiac hypertrophy by directing glucose to aspartate biosynthesis. *Circulation Research*.

[151] Yu Z., Chen R., Li M. (2018). Mitochondrial calcium uniporter inhibition provides cardioprotection in pressure overload-induced heart failure through autophagy enhancement. *International Journal of Cardiology*.

[152] Wang B., Nie J., Wu L. (2018). AMPK*α*2 protects against the development of heart failure by enhancing Mitophagy via PINK1 phosphorylation. *Circulation Research*.

[153] Laker R. C., Drake J. C., Wilson R. J. (2017). Ampk phosphorylation of Ulk1 is required for targeting of mitochondria to lysosomes in exercise-induced mitophagy. *Nature Communications*.

[154] Gwinn D. M., Shackelford D. B., Egan D. F. (2008). AMPK phosphorylation of raptor mediates a metabolic checkpoint. *Molecular Cell*.

[155] Egan D. F., Shackelford D. B., Mihaylova M. M. (2011). Phosphorylation of ULK1 (hATG1) by AMP-activated protein kinase connects energy sensing to mitophagy. *Science*.

[156] Liao H., Gao W., Ma J. (2021). GPR39 promotes cardiac hypertrophy by regulating the AMPK–mTOR pathway and protein synthesis. *Cell Biology International*.

[157] Toyama E. Q., Herzig S., Courchet J. (2016). Metabolism. AMP-activated protein kinase mediates mitochondrial fission in response to energy stress. *Science*.

[158] Zhang T., Chi Y., Kang Y. (2019). Resveratrol ameliorates podocyte damage in diabetic mice via SIRT1/PGC-1*α* mediated attenuation of mitochondrial oxidative stress. *Journal of Cellular Physiology*.

[159] Lee I. H., Cao L., Mostoslavsky R. (2008). A role for the NAD-dependent deacetylase Sirt1 in the regulation of autophagy. *Proceedings of the National Academy of Sciences of the United States of America*.

[160] Jang S. Y., Kang H. T., Hwang E. S. (2012). Nicotinamide-induced Mitophagy:. *The Journal of Biological Chemistry*.

[161] Das S., Mitrovsky G., Vasanthi H. R., Das D. K. (2014). Antiaging properties of a grape-derived antioxidant are regulated by mitochondrial balance of fusion and fission leading to mitophagy triggered by a signaling network of Sirt1-Sirt3-Foxo3-PINK1-PARKIN. *Oxidative Medicine and Cellular Longevity*.

[162] Dong H. W., Zhang L. F., Bao S. L. (2018). AMPK regulates energy metabolism through the SIRT1 signaling pathway to improve myocardial hypertrophy. *European Review for Medical and Pharmacological Sciences*.

[163] Ou X., Lee M. R., Huang X., Messina-Graham S., Broxmeyer H. E. (2014). SIRT1 positively regulates autophagy and mitochondria function in embryonic stem cells under oxidative stress. *Stem Cells*.

[164] Liang D., Zhuo Y., Guo Z. (2020). SIRT1/PGC-1 pathway activation triggers autophagy/mitophagy and attenuates oxidative damage in intestinal epithelial cells. *Biochimie*.

[165] Brainard R. E., Facundo H. T. (2021). Cardiac hypertrophy drives PGC-1*α* suppression associated with enhanced O-glycosylation. *Biochimica et Biophysica Acta - Molecular Basis of Disease*.

[166] Chen C. Y., Chen J., He L., Stiles B. L. (2018). PTEN: tumor suppressor and metabolic regulator. *Frontiers in endocrinology*.

[167] Cai J., Li R., Xu X. (2018). CK1*α* suppresses lung tumour growth by stabilizing PTEN and inducing autophagy. *Nature Cell Biology*.

[168] Li M., Yang X., Wang S. (2018). PTEN enhances nasal epithelial cell resistance to TNF*α*-induced inflammatory injury by limiting mitophagy via repression of the TLR4-JNK-Bnip3 pathway. *Molecular Medicine Reports*.

[169] Li P., Wang J., Zhao X. (2020). PTEN inhibition attenuates endothelial cell apoptosis in coronary heart disease via modulating the AMPK–CREB–Mfn2-mitophagy signaling pathway. *Journal of Cellular Physiology*.

[170] Chen C., Zou L. X., Lin Q. Y. (2019). Resveratrol as a new inhibitor of immunoproteasome prevents PTEN degradation and attenuates cardiac hypertrophy after pressure overload. *Redox Biology*.

[171] Tian M., Jiang X., Li X., Yang J., Zhang C., Zhang W. (2021). LKB1IP promotes pathological cardiac hypertrophy by targeting PTEN/Akt signalling pathway. *Journal of Cellular and Molecular Medicine*.

[172] Hoshino A., Mita Y., Okawa Y. (2013). Cytosolic p53 inhibits Parkin-mediated mitophagy and promotes mitochondrial dysfunction in the mouse heart. *Nature Communications*.

[173] Guo J., Mihic A., Wu J. (2015). Canopy 2 attenuates the transition from compensatory hypertrophy to dilated heart failure in hypertrophic cardiomyopathy. *European Heart Journal*.

[174] Xiao L., Xu X., Zhang F. (2017). The mitochondria-targeted antioxidant MitoQ ameliorated tubular injury mediated by mitophagy in diabetic kidney disease via Nrf2/PINK1. *Redox Biology*.

[175] Gureev A. P., Sadovnikova I. S., Starkov N. N., Starkov A. A., Popov V. N. (2020). p62-Nrf2-p62 Mitophagy regulatory loop as a target for preventive therapy of neurodegenerative diseases. *Brain Sciences*.

[176] Tang C., Yin G., Huang C. (2020). Peroxiredoxin-1 ameliorates pressure overload-induced cardiac hypertrophy and fibrosis. *Biomedicine & Pharmacotherapy*.

[177] Kamo T., Akazawa H., Komuro I. (2015). Cardiac nonmyocytes in the hub of cardiac hypertrophy. *Circulation Research*.

[178] Tian G., Zhou J., Quan Y., Kong Q., Wu W., Liu X. (2021). P2Y1 receptor agonist attenuates cardiac fibroblasts activation triggered by TGF-*β*1. *Frontiers in Pharmacology*.

[179] Schimmel K., Ichimura K., Reddy S., Haddad F., Spiekerkoetter E. (2022). Cardiac fibrosis in the pressure overloaded left and right ventricle as a therapeutic target. *Frontiers in Cardiovascular Medicine*.

[180] Gibb A. A., Lazaropoulos M. P., Elrod J. W. (2020). Myofibroblasts and fibrosis: mitochondrial and metabolic control of cellular differentiation. *Circulation Research*.

[181] Guan C., Zhang H. F., Wang Y. J. (2021). The downregulation of ADAM17 exerts protective effects against cardiac fibrosis by regulating endoplasmic reticulum stress and mitophagy. *Oxidative Medicine and Cellular Longevity*.

[182] Zhang Y., Wang Z., Lan D. (2022). MicroRNA-24-3p alleviates cardiac fibrosis by suppressing cardiac fibroblasts mitophagy via downregulating PHB2. *Pharmacological Research*.

[183] Ren Z., Yu P., Li D. (2020). Single-cell reconstruction of progression trajectory reveals intervention principles in pathological cardiac hypertrophy. *Circulation*.

[184] Yang D., Liu H. Q., Liu F. Y. (2021). Critical roles of macrophages in pressure overload-induced cardiac remodeling. *Journal of Molecular Medicine*.

[185] Revelo X. S., Parthiban P., Chen C. (2021). Cardiac resident macrophages prevent fibrosis and stimulate angiogenesis. *Circulation Research*.

[186] Patoli D., Mignotte F., Deckert V. (2020). Inhibition of mitophagy drives macrophage activation and antibacterial defense during sepsis. *The Journal of Clinical Investigation*.

[187] Dittrich G. M., Froese N., Wang X. (2021). Fibroblast GATA-4 and GATA-6 promote myocardial adaptation to pressure overload by enhancing cardiac angiogenesis. *Basic Research in Cardiology*.

[188] Wei T., Huang G., Gao J. (2017). Sirtuin 3 deficiency accelerates hypertensive cardiac remodeling by impairing angiogenesis. *Journal of the American Heart Association*.

[189] Tan Y., Li M., Wu G. (2021). Short-term but not long-term high fat diet feeding protects against pressure overload-induced heart failure through activation of mitophagy. *Life Sciences*.

[190] Ito Y., Maejima Y., Tamura N. (2018). Synergistic effects of HMG-CoA reductase inhibitor and angiotensin II receptor blocker on load-induced heart failure. *FEBS Open Bio*.

[191] Chen X., Jiang X., Cheng C. (2020). Berberine attenuates cardiac hypertrophy through inhibition of mTOR signaling pathway. *Cardiovascular Drugs and Therapy*.

[192] Liu B. Y., Li L., Liu G. L. (2021). Baicalein attenuates cardiac hypertrophy in mice via suppressing oxidative stress and activating autophagy in cardiomyocytes. *Acta Pharmacologica Sinica*.

[193] Zhao W., Li Y., Jia L., Pan L., Li H., du J. (2014). Atg5 deficiency-mediated mitophagy aggravates cardiac inflammation and injury in response to angiotensin II. *Free Radical Biology & Medicine*.

